RETRACTED

# Renewable energy, regional tourism, and exports to tackle stagnant growth in developed economies

**DOI:** 10.1016/j.heliyon.2024.e37190

**Published:** 2024-09-03

**Authors:** Hunag Chenhui, Muhammad Shahid Hassan, Sahar Afshan, Imran Hanif, Muhammad Umair, Olayan Albalawi

**Affiliations:** a Wenzhou Vocational and Technical College, Wenzhou, Zhejiang, 325000, China; b Department of Economics and Quantitative Methods, Dr. Hassan Murad School of Management (HSM), University of Management and Technology Lahore, Pakistan; c Department of Economics and Finance, Sunway Business School, Sunway University, Subang Jaya, Malaysia; d Department of Economics, Government College University Lahore, Pakistan; e Adnan Kassar School of Business, Lebanese American University, Beirut, Lebanon; f Department of Economics, Ghazi University, Dera Ghazi Khan, Pakistan; g Western Caspian University, Baku, Azerbaijan; h Department of Statistics, Faculty of Science, University of Tabuk, Tabuk, Saudi Arabia; i Department of Economics, Korea University, Seoul, South Korea

**Keywords:** Foreign direct investment, Regional tourism, Renewable energy, CS-ARDL, Stagnant growth

## Abstract

This study examines the effects of energy resources in the form of clean and unclean energy on the economic progress of 30 selected developed economies. This study used data from 1990 to 2020 and it employs the CS-ARDL method to obtain results. The results present that both clean and unclean energy significantly stimulate economic progress. The findings further expose that foreign investment resources in the form of inflow are significant factors that accelerate economic progress in developed economies. The results reveal that tourism development, capital accumulation, and exports are significant factors in boosting economic progress in the selected economies. Estimates from Dumitrescu and Hurlin's method for heterogeneous panels confirm the presence of the feedback-effect hypothesis for unclean energy, while the energy-conservation hypothesis holds for clean energy. This study suggests that targeting low-cost clean energy production is crucial for promoting economic growth and protecting the environment through carbon mitigation strategies. There is also a need to develop a policy framework that emphasizes the transformation of industry towards clean energy at a macro level. Furthermore, transitioning from unclean to clean energy may enhance economic progress by improving environmental quality norms in the selected developed economies. Finally, policies for tourism development, export improvement, and increased inflow of FDI should be directed towards fostering clean energy agreements and achieving environment-friendly economic progress in developed economies.

RETRACTED

## 1 Introduction

Energy has earned an imperative position in the production function in both developed and developing economies. As far as its impact on production is concerned, it is inconclusive. In some economies, it significantly elevates production activities as stated by Ren et al. [1] while the various energy generation methods leave a significant adverse influence on environmental quality at the global level [2]. Besides this, the use of energy still seems an insignificant attribute to the upward shift of production function, as compared to other economic factors [3]. However, to highlight the energy-growth relationship a variety of studies have performed causality analysis to explain the four fundamental hypotheses. For instance, the Neutrality-Hypothesis advocates no causality between the use of energy and economic progress [4]. The growth hypothesis mentioned a causal relationship between energy utilization to improved economic progress, according to Hazarik [5]. The Conservation Hypothesis or Growth-Led-Energy Hypothesis states a direction of causal association from high growth to high energy use stated by Bekun and Agboola [6]. Finally, the Bidirectional-Causal-Relation represents that both energy and growth cause each other, as stated by Satti et al. [7]. There are also such types of studies in which renewable has been witnessed to significantly lift economic progress [[8], [9]]. Unlike clean energy, the effect of unclean energy is also witnessed as positive on economic progress [10]. Contrarily, Ozturk et al. [11] disclosed that the high consumption of clean energy suppresses economic progress. Based on this discussion, in our study, we also considered energy as input for targeting production activities among the developed economies. From a theoretical perspective, the impact of renewable energy or clean energy on economic growth may provide multiple channels. If the expenditures on clean or green energy are enhanced it tends to encourage competitiveness through achieving economies of scale. Hence it deteriorates energy costs and improves infrastructure development in the country. This helps in improving domestic production and hence leads to economic growth. It is further intuited that the reliance on clean energy helps in creating numerous jobs by stimulating local economies. This is a labor-intensive sector and during the installation and maintenance phase, more labor is required hence it leads to more employment creation. The increased supply of labor tends to improve domestic output or increase economic growth. Salehin and Kiss [12] suggested that economic growth was improving due to expansion in renewable energy in 15 emerging countries while similar results were highlighted by Kahia et al. [13] in the case of net oil-importing economies from the MENA region. The contribution of Esposito [14] and Mohamed et al. [15] reported a feedback effect between renewable energy and economic growth while Hung-Pin [16] disclosed that economic growth was strongly caused by renewable energy in the long run in cases of Germany and the UK. Afterward, Alhasim et al. [17] highlighted the linear but positive impact of clean energy on the output of E−7 economies. These studies have motivated us to consider the role of renewable energy to capture its effects on domestic output in our study hence we have taken it as a driver of economic growth.

RETRACTED

While inquiring about the drivers of economic progress in the literature, we find so many studies in which primary and important inputs such as labor force and capital formation are ignored [7]. From the history of the production function, it is always considered an obligation to augment the production function by at least considering two basic inputs such as capital and labor [[8], [18], [19], [20]]. Along with the basic factors of production function, Isik et al. [21] considered governance, environmental, and social indicators to develop a relationship with economic growth in South Asia and the East Asia Pacific. In another study, Isik et al. [22] considered governance, environmental, and social indicators to develop a relationship with sustainable development goals in BRIC-11 nations.

At the current time, tourism development is getting attention to be considered an essential actor for stimulating production activities in any economy [[23], [24]]. The possible impact of tourism development on economic progress can help policymakers consider tourism as part of their policy function while targeting economic progress [[25], [26], [27]]. As the inflow of foreign exchange from expansion in tourism enhances then it will surely give a boost to economic activities in any economy according to Rehman et al. [28], Rasool et al. [29], and Sokhanvar and Jenkins [30]. This discussion has motivated us to take tourism development as an input in our production function. Moreover, from a theoretical perspective, tourism may be considered an important driver of economic growth. Tourism invites foreigners who bring foreign exchange with them. This extends earnings in the form of foreign exchange on the one side and the tourists also tend to promote local business activities. This entire process helps improve the balance of payment, reduces regional disparities, escalates domestic employment, develops physical infrastructure, and above all promotes domestic production in the country. The empirical study of Aini [31] for 15 Southeast Asian countries reported a significantly positive role of tourism on economic growth. Haini et al. [32] suggested that tourism through a strong institutional set up helped in promoting economic growth in 143 economies. Afterward, we find Sarkhanov and Baghirov [33] who validated the tourism-led-growth hypothesis for Ukraine; Georgia, Azerbaijan, and Moldova countries. Based on this discussion, this research considered the significance of tourism development in promoting economic growth of the countries and hence has taken tourism as a driver of economic growth. From a theoretical perspective, the expansion of exports allows efficient utilization of resources and hence promotes specialization in the country. It further helps in exploring new methods of production, motivates to use of modern technology and all this ultimately helps in expanding domestic production. Therefore, economic growth expands. The direct impact of exports on economic growth was witnessed by Kim and Seok [34] for the Korean economy and Ahmad et al. [35] for the Singapore case. Besides this, the increasing behavior of trade liberalization to stimulate economic growth was found by Jabbar et al. [36] in Luxembourg while Riaz et al. [37] suggested the same results for Portugal's economy. Based on this discussion, this study takes into account the “Export-led-Growth” hypothesis to investigate whether it is relevant in the selected economies. During the period of globalization, trade liberalizing bodies circulated the notion of the promotion of free trade around the globe. This notion has highlighted the pivotal role of exports and the inflow of FDI via which the progress of any economy can be stimulated [[38], [39]].

RETRACTED

Both FDI and exports are helpful in significantly promoting domestic output [35. 36]. The literature reveals our attention to the Export-Led Growth Hypothesis-which states that the expansion of exports encourages production-related activities in the country [[40], [41]]. The effects of the FDI inflow are inconclusive. For instance, Ciobanu [42] highlighted the insignificant role of FDI in economic progress while Olayungbo and Quadri [[43], [44]] and Appiah et al. [45] suggested that it has an adverse influence on economic progress. However, Kalai and Zghidi [[46], [47]]and Worku [48] presented FDI as a booster of economic progress.

Based on the discussion above, it is crucial to differentiate between clean and unclean energy to reveal their respective contributions to economic progress. This study also considers key factors such as tourism development, exports, and inflow of FDI to examine their potential effects on the economic progress of the selected developed economies. (a) The primary objective of the study is to investigate how clean energy or renewable energy may foster economic growth in developed economies. (b) The second objective is to uncover how the tourism industry can improve economic growth. (c) The third objective is to spotlight how exports and FDI inflow could influence the economic progress of developed nations. This study is unique in its approach, as we have found few studies that jointly determine the effects of tourism development, exports, and FDI inflow, along with renewable and unclean energy, on economic progress using a production function approach in a panel study.

Therefore, to make our work innovative, we introduced energy, tourism, and export variables into our production function to adhere to the assumptions of the production function approach. In addition to these primary inputs, we will enhance our production function by including the aforementioned significant drivers of economic progress. Thus the primary research problem addressed is understanding the specific mechanisms through which renewable energy, tourism, and foreign trade drive economic growth. The paper explores the underlying mechanisms, interdependencies, and synergies between these sectors, and provides evidence-based policy recommendations. It offers a comprehensive and actionable understanding of how these sectors can be strategically developed to combat stagnant growth and promote sustainable economic development.

The paper synthesizes theoretical arguments and empirical evidence on the roles of renewable energy, tourism, and foreign trade in combating stagnant economic growth by analyzing 30 developed economies. The findings reveal that foreign investment inflows are significant in accelerating economic progress. Tourism development, capital accumulation, and exports are also critical factors in boosting economic growth. The study confirms the feedback-effect hypothesis for unclean energy and the energy-conservation hypothesis for clean energy, suggesting that low-cost clean energy production is crucial for promoting economic growth and protecting the environment through carbon mitigation strategies. Innovatively, the paper adopts a holistic approach, examining the synergies between renewable energy, tourism, and foreign trade rather than analyzing them in isolation. It highlights how developments in one sector can positively impact others and proposes a new analytical framework for evaluating the potential impacts of investments in these sectors on economic growth. The paper emphasizes the need to develop a policy framework that promotes the transformation of industry towards clean energy at a macro level. Transitioning from unclean to clean energy is essential for enhancing economic progress and improving environmental quality norms. Additionally, this study employs the CS-ARDL method, the most recent methodology for heterogeneous panels, to capture reliable and significant results. From a policy perspective, this study is important for the selected developed economies as it provides insights into the roles of unclean and clean energy in fostering economic progress, considering other significant economic factors such as tourism development, exports, and FDI inflow, through the use of a production function.

RETRACTED

In the second section, a brief discussion is presented to highlight some factors that may influence economic progress. In section 3, sources of data, the composition of the model, and methods will be highlighted. Results will be estimated in section 4 and the conclusion will be given in section 5.

## 2 Literature review

To establish a precise relationship between clean energy, exports, FDI inflow, and tourism development with economic progress it is essential to review the literature to establish a foundation for research study, building a literature gap and appropriate research design.

### 2.1 Review of empirical studies

The studies have inquired about the use of clean energy in targeting economic progress. From the contribution of Kocak and Sarkgunesi [49], we may see that they utilized FMOLS and DOLS estimators to analyze panel data and depicted the positive influence of renewable energy on the economic progress of the Black Sea and Balkan nations. Haseeb et al. [50] considered the ARDL approach and depicted that economic progress was enhanced significantly with the use of renewable energy in Malaysia. Besides that, Qudrat-Ullah and Nevo [51] used the GMM estimation method to analyze data and depicted that renewable energy consumption promotes economic progress, while the labor force influenced economic progress insignificantly in the selected 37 African economies. After employing fixed effect methods by considering data from 1990 to 2014, Akram et al. [52] concluded an adverse impact of clean energy on output in the selected BRICS economies. The study further reported estimates of quantile regression in which the coefficient of capital formation was turned negative instead of positive. The impact of nonrenewable energy on economic progress was tested by many scholars in their research. As we see Satti et al. [7] considered causality analysis and confirmed a two-way association of nonrenewable energy and economic progress in Pakistan. Khan et al. [53] determined the impact of renewable energy on carbon emissions and economic development in SAARC nations, accounting for geographical variability. Findings depicted that clean energy is a key factor for carbon neutrality, especially in higher quantiles. The study suggests following a balanced and environment-friendly growth path by taking the initiative of increasing renewable energy share. Okumus and Kocak [54] developed theoretical, practical, and political implications to establish a linkage between economic growth and tourism. They confirmed tourism as a significant indicator to promote growth in the United States. Moreover, effects of the expansion and contraction of the tourism industry in the US are asymmetrical. Ashfaq et al. [55] elaborated that green economic growth and economic globalization improve the usage of clean energy in the long-term period. They further exposed that a high share of renewable energy consumption in total energy has not reduced emissions in industrialized countries. After applying the Johansen approach to analyze data from 1977 to 2013, Hassan et al. [56] concluded the significantly accelerating role of natural gas consumption as a proxy for nonrenewable energy upon economic progress in Pakistan. There are many studies conducted by scholars across the world who have captured the influence of clean energy and nonrenewable energy upon economic progress by considering the production function approach. For instance, Pao et al. [57] reported a significantly elevating response of economic progress toward energy and capital stock. The study also reported a negative influence of the labor force on economic progress in the selected four MIST economies. According to Bhattacharya et al. [58] the estimates of FMOLS and DOLS depict a positive influence of clean and unclean energy use on economic progress in the top 38 selected economies. Ji and Yang [59] highlighted that renewable energy helps to control carbon emissions. Moreover, they mentioned that tourism development and the digital economy are the key factors to promote green growth in BRICS nations. Liue et al. [60] found a two-way linkage between renewable energy and output, while one-way association from trade to output. Mohamed et al. [15] explored the dynamic relationship between tourism, trade, economic progress, and carbon release by analyzing panel data from central and South American nations. They found that economic progression and trade both contribute to carbon release, while renewable energy, tourism development, and FDI are helping to reduce carbon release in the long run period. The study conducted by Amri [61] applied the bounds test to data from 1980 to 2012 and concluded that both capital stock and unclean energy significantly expanded economic progress while renewable energy remained an insignificant determinant of economic progress in Algeria. Later on, the significantly boosting role of energy consumption was found by Kahia et al. [13] by utilizing the FMOLS estimator over the period from 1980 to 2012 for the MENA economies. According to Ntanos et al. [62], the results of the ARDL for the sample period from 2007 to 2016 confirmed a significantly escalating response of economic progress toward an increase in energy use in 25 selected European economies. Gozgor et al. [63] employed a panel ARDL and reported a significant positive influence of energy on economic progress in OECD nations. Afterward, the estimates of panel GMM techniques for BRICS countries confirmed the significant roles of capital stock, labor force, and nonrenewable energy in expanding economic progress. The results further disclosed that renewable energy remained an insignificant driver of economic progress in the selected BRICS countries [64]. Besides this, we see Singh et al. [65] conducted a study in which they employed FMOLS by considering developing and developed economies data from 1995 to 2016 and exposed that labor force, capital formation, and energy production left positive and significant effects on economic progress in the selected sample economies. After that, Le et al. [66] utilized the GMM technique by considering the data range from 1996 to 2012 and depicted a positive association of energy resources with economic progress in the selected sample of 102 economies. Through the bounds test the positive role of energy to foster economic progress was also disclosed by Pegkas [67] for Greece's economy.

RETRACTED

Rehman et al. [68] investigated the influence of various exports and foreign investments on Pakistan's economic progress from 1976 to 2019 with the NARDL method. Short-term findings indicate diverse effects: communication technology exports demonstrate both positive and negative impacts, while exports and services negatively affect economic progress. Foreign investment unveils dual effects. Long-term outcomes expose similar patterns, with foreign investment presenting an adverse impact, and goods, services, and food exports having a negative effect. Manufacturing exports depicted a steadily negative effect on economic growth in both periods. Rehman et al. [69] use an asymmetric ARDL model to examine the impacts of various economic factors on Pakistan's growth from 1976 to 2019. Total reserves negatively but insignificantly affect growth. Positive shocks in remittances positively stimulate growth. Positive shocks in gross savings are favorable but insignificant, and positive shocks in FDI are detrimental. Finally, better infrastructure policies employing foreign investment are recommended. Deng et al. [70] utilized a holistic index and advanced econometric techniques, they found a long-term relationship and threshold effects. According to the findings, FDI initially reduces, then increases pollution, with different patterns across income groups. Financial development and social globalization consistently increase pollution. Policy implications emphasize achieving UN Sustainable Development Goals. Halilbegović et al. [71] employed advanced panel estimation techniques, they determined that energy either renewable or conventional both positively affect economic growth. The study suggests prioritizing investment in clean energy projects to support sustainable growth.

RETRACTED

Rehman et al. [72] analyze the role of financial development and political stability in adopting renewable energy in 17 emerging economies from 1994 to 2021. They find that environmental taxes promote renewable energy adoption, while political stability and financial development provide necessary support. These results can inform policies to facilitate sustainable energy transitions. Rehman et al. [73] employed the NARDL technique and found that negative globalization and growth shocks have mixed effects on carbon release, higher population growth increases emissions, and renewable energy has no significant impact. Nuclear energy consumption reduces emissions. Recommendations include new strategies to reduce global carbon emissions. Rehman et al. [74] studied the impact of various energy sources and urbanization on Romania's economic development using ARDL, FMOLS, and CCR techniques. They found that energy from fuels and nuclear fusion positively affect growth. Policies addressing energy consumption are needed for economic improvement. Işık et al. [75] propose new determinants for environmental pollution models, focusing on the USA. They introduce the domestic-exports/re-exports ratio and climate policy uncertainty index, finding that increased re-exports reduce CO2 emissions, while climate policy uncertainty does not affect emissions. These new determinants can help policymakers better understand trade patterns' environmental impact.

In a study, we see Fu et al. [76] used DOLS and FMOLS and DOLS and depicted energy and economic progress are positively correlated in the BRICS economies. Later on, Syzdykova et al. [77] employed a GMM estimator by taking a sample from 1990 to 2019 and showed a positive influence of energy on economic progress. From the contribution of Asiedu et al. [10], we see that the estimates of DOLS and FMOLS for the sample from 1990 to 2018 demonstrated that both clean and unclean energy were found to significantly stimulate economic progress in the selected 26 European economies. After utilizing panel OLS, DOLS, FMOLS, and fixed effect estimators over the sample from 1995 to 2017, a study by Asif et al. [78] concluded that clean energy and unclean energy were significantly expanding economic progress in the selected 99 economies.

RETRACTED

In a recent study conducted by Ozturk et al. [11], they considered data ranging from 1991 to 2016 and depicted significant negative effects of renewable energy on economic progress while the labor force was found to significantly boost economic progress in the selected 20 economies. Wang et al. [79] applied a bound test to analyze the data from 1980 to 2019 and found a U-shaped association between renewable energy and the inverted U-shaped impact of nonrenewable energy on economic progress. The findings confirmed the significant boosting impact of the export value index on economic progress for Pakistan. In another study, Hassan et al. [80] after employing the NARDL approach over the period from 1972 to 2019 demonstrated appreciating and significant effects of electricity use on economic progress.

The literature has also highlighted the role of tourism development in promoting the economic activities of any country. Therefore, we consider the conducted of Bulgan et al. [23] examined the influence of tourism on the economic progress of the Turkish economy. They determined tourism development has the potential to improve economic progress by applying the ARDL bound test method. Afterward, we find Rehman et al. [28] who tested the impact of tourism expenditures on the economic progress of Pakistan's economy. They employed bounds testing and inferred a positive and significant influence of all three proxies of tourism expenditures on economic progress for Pakistan. Moreover, the impact of tourism development and the inflow of FDI in tourism and non-tourism sectors on economic progress was tested by Menyari [25]. The bounds test results inferred a positive influence of tourism on economic progress while the inflow of FDI in the tourism sector was reducing economic progress. While in the non-tourism sector, an inflow of FDI was significantly enhancing economic progress in Morocco. After employing a PMG estimator on data from 1995 to 2015, Rasool et al. [29] disclosed that tourism development significantly enhanced economic progress in BRICS economies. Besides them, Sokhanvar and Jenkins [30] examined how changes in FDI and international tourism development are changing economic progress in Estonia. After utilizing the NARDL estimator over the period from 1995 to 2019, this study confirms the significantly appreciating impact of FDI on economic progress in Estonia. Wu et al. [26] applied a quantile-on-quantile method to Eastern China's data from 1995 to 2020 and reported a significant contribution of tourism to foster economic progress.

RETRACTED

There are many pieces of research available that highlight the export-led growth hypothesis. Haseeb et al. [38] inquired about the role of exports and FDI in targeting the economic progress of the Malaysian economy. They applied the bounds testing method and reported a significantly positive association between exports, FDI, and economic progress in Malaysia. Besides them, Ahmad et al. [81] conducted research in which they applied the ARDL bounds test to analyze data from 1972 to 2014 and established an export-led growth hypothesis for Pakistan. The study made by Sultanuzzaman et al. [82] also considered the bounds testing approach and depicted the positive influence of inflows of FDI on economic progress. Moreover, exports significantly hamper economic progress in the long-run period while in the short-run period, economic progress is enhanced due to an increase in exports of Sri Lanka. Afterward, we see Canbay [40] who executed research for testing the influence of exports on the economic progress of Turkey. The application of the bounds test for the data series from 1989 to 2016 reported the validation of the export-led growth hypothesis for Turkey. In another research, we find Logun [83] who inquired about the impact of exports and FDI for seven emerging economies by applying the ARDL method. The study inferred that FDI and exports significantly expand economic progress only in the long run in the selected seven emerging economies.

The researchers also revealed attention to an important driver of economic progress in their research and it is FDI. According to Olayungbo and Quadri [43], the estimates of the panel ARDL technique over the sample from 2000 to 2015 inferred that FDI significantly reduced economic progress over the long run period while it significantly enhanced economic progress in the short run in sub-Saharan African economies. For a similar period, Appiah et al. [45] also applied the panel ARDL method over the period from 1995 to 2015 and disclosed a significantly positive influence of FDI on economic progress while the labor force reduces economic progress in five selected African countries. The contribution by Kalai and Zghidi [46] considered the panel ARDL approach and inferred that FDI and capital formation left significantly escalating effects on economic progress while the labor force exposed an insignificant impact on economic progress in the selected 15 MENA countries. Afterward, Ciobanu [42] considered the annual data series from 1991 to 2018 and applied the bounds test that showed an insignificant impact of FDI on the economic progress of the Romanian economy. In a study, we see Worku [48] who employed random effect, DOLS, and panel ARDL to estimate data from 1975 to 2019 and concluded that economic progress responded positively due to an increase in the inflow of FDI in the selected nine East African economies.

RETRACTED

### 2.2 Theoretical background

After reviewing the literature section in detail, we have framed our function forms based on a theoretical foundation. The study used a Solow growth model to obtain the objectives of this study. Thus, by following the Solow growth model the functional form of the study is given in Equation (1);

(1) Output=f(Labor,Capital,Technology)

Following the above functional form, the studies of Pao et al. [57], Bhattacharya et al. [58], Kahia et al. [13], and Asif et al. [78] considered an output function by considering two primary inputs such as labor force and capital stock along with energy in their studies. This has motivated us to consider primary inputs in the production function. Besides this, Satti et al. [7] and Hassan et al. [56] considered coal consumption and natural gas consumption as proxies for nonrenewable energy as inputs to economic progress while Singh et al. [65], Le et al. [66], Asiedu et al. [10], Fu et al. [76], Syzdykova et al. [77], Wang et al. [79] considered energy as input in a production function to access economic progress in their studies. We have also considered energy as input in production functions to see how they would respond to our selected sample. Afterward, when we reviewed the contribution of Bulgan et al. [23], Rehman et al. [28], Menyari [25], Rasool et al. [29], Sokhanvar and Jenkins [30], and Wu et al. [26], then we feel convenient to consider international tourism as a determinant of economic progress in our study. Beyond doubts, the research of Haseeb et al. [38], Ahmad et al. [81], Sultanuzzaman et al. [82], Canbay [40], and Logun [83] have motivated us to consider export as an important input for testing its impact on production activities. Therefore, we have taken exports as an input to economic progress in our study. This will guide us to inquire about the presence or absence of export-led growth in our study. For the last factor, the research studies of Olayungbo and Quadri [43], Appiah et al. [45], Kalai and Zghidi [46], Ciobanu [42], and Worku [48] have guided us that FDI can be considered as an important factor that can also help in leaving spillover effects on production activities. Therefore, this has allowed us to consider FDI as an important determinant of economic progress in our study.

RETRACTED

Based upon the above-reviewed literature, we find it suitable to consider energy, tourism development, exports, and FDI in a production function given in Equation (1). In the next section, the data source, model, and methodological framework will be discussed in detail.

## 3 Data source and estimation strategy

The present study considers a second sample for the annual data series from 1990 to 2020 for the selected 30 developed economies (list attached in Appendix-1). The data on all the variables are collected from the World Bank [84]. Moreover, the purpose of selecting developed nations for econometric analysis is based on data availability, particularly the data on tourism development and export indicators. Thus the study considered 30 industrialized nations with possible maximum duration to attain the objectives of the study. In this study, we propose the functional forms given in Equation (2) and Equation (3) for obtaining empirical results.

(2) $${\text{lnGDPPC}}_{\text{it}}=f\;\left({\text{lnLAB}}_{\text{it}},{\text{lnCAP}}_{\text{it}},{\text{lnTOUR}}_{\text{it}},{\text{lnFFEC}}_{\text{it}},{\text{lnREC}}_{\text{it}},{\text{lnEXPORT}}_{\text{it}}\right)$$

(3) $${\text{lnGDPPC}}_{\text{it}}=f\;\left({\text{lnLAB}}_{\text{it}},{\text{lnCAP}}_{\text{it}},{\text{lnTOUR}}_{\text{it}},{\text{lnFFEC}}_{\text{it}},{\text{lnREC}}_{\text{it}},{\text{lnFDI}}_{\text{it}}\right)$$

Here, brief descriptions of dependent and independent variables are given in Table 1.

**Table – 1:** Variables descriptions.

**Variables**	**Names**	**Transformation**	**Source**
${\text{lnGDPPC}}_{\;\text{it}}$	Per Capita Economic Growth	$\begin{array}{l} {\text{lnGDPPC}}_{\text{it}}=\\ \ln\;\left[{\text{GDP}}_{\text{it}}\;/\;{\text{Population}}_{\text{it}}\right] \end{array}$	World Bank (2022)
${\text{lnLAB}}_{\text{it}}$	Total Labor Force	$\begin{array}{l} {\text{lnLAB}}_{\;\text{it}}=\\ \ln\;\left[\text{Total}\;\text{Labor}\;{\text{Force}}_{\;\text{it}}\right] \end{array}$	World Bank (2022)
${\text{lnCAP}}_{\text{it}}$	Gross Fixed Capital Formation as a share of GDP	$\begin{array}{l} {\text{lnGFCF}}_{\text{it}}=\\ \ln\;\left[{\text{GFCF}}_{\text{it}}\;/\;{\text{GDP}}_{\text{it}}\right] \end{array}$	World Bank (2022)
${\text{lnTOU}}_{\text{it}}$	International Tourism, Number of Arrivals	$\begin{array}{l} {\text{lnTOUR}}_{\text{it}}=\\ \ln\;\left[{\text{Number}\;\text{of}\;\text{Arrivals}}_{\text{it}}\;\right] \end{array}$	World Bank (2022)
${\text{lnFFEC}}_{\;\text{it}}$	Fossil Fuel Energy use (% of total energy use)	$\begin{array}{l} {\text{lnFFEC}}_{\;\text{it}}=\ln\;[\text{FFEC}\;\text{it}\;/\\ \text{Total}\;\text{Energy}\;] \end{array}$	World Bank (2022)
${\text{lnREC}}_{\;\text{it}}$	Renewable Energy Output (% of total Output)	$\begin{array}{l} {\text{lnREC}}_{\;\text{it}}=\\ \ln\;\left[\text{REC}\;\text{it}\;/\;\text{Total}\;\text{Output}\;\text{it}\;\right] \end{array}$	World Bank (2022)
${\text{lnEXPORT}}_{\;\text{it}}$	Exports as a share of GDP	$\begin{array}{l} {\text{lnEXPORT}}_{\;\text{it}}=\\ \ln\;\left[\text{EXPORT}\;\text{it}\;/\;\text{GDP}\;\text{it}\;\right] \end{array}$	World Bank (2022)
${\text{lnFDI}}_{\;\text{it}}$	FDI as a share of GDP (Net Inflows)	${\text{lnFDI}}_{\;\text{it}}=\ln\;\left[\text{FDI}\;\text{it}\;/\;\text{GDP}\;\text{it}\;\right]$	World Bank (2022)

The above-stated variables in the functional form are computed using the log transformation approach. This approach provides more efficient and reliable estimates than the non-log transformation approach. It is convenient to interpret and compare results across other studies by Yu-Ke et al. [85], Hassan et al. [86], Kalim and Hassan [87], and Mahmood et al. [88]. To estimate empirical results, the present study will follow the following structure.

RETRACTED

To identify a significant correlation between explanatory variables, we will apply the variance inflation factor by using Equation (4). If the value of the VIF test exceeds or turns equal to ten, then it will depict a severe multicollinearity issue.

(4) $$\text{VIF}=\frac{1}{1\;-\;{\left(r_{\text{xy}}\right)}^{2}}$$

Pesaran [89] presented Equation (5) for diagnosing CD in the data series. The null hypothesis of no CD will be rejected if the probability value of the test exceeds or becomes equal to 10 percent.

(5) $$\text{CD}=\sqrt{\frac{2T}{N\;\left(N-1\right)}}\;\left(\sum_{i=1}^{N\;-\;1}\sum_{j=i+1}^{N}\;{\hat{\rho }}_{\text{ij}}\right)\;\Rightarrow \;N\;\left(0,1\right)$$

The contribution of Pesaran [90] guides the application of CIPS and CADF unit root tests in the presence of CD issues. Equation (6) and Equation (7) represent the generalized form of CIPS and CADF tests respectively.

(6) $$\text{CIPS}\;\left(N,T\right)=N^{-1}\;\sum_{i=1}^{N}\;t_{i}\;\left(N,T\right)$$

(7) $$\text{CADF}{\;}_{i\int }=\frac{\int_{0}^{1}W_{i}\;\left(r\right)\;d\;W_{i}\;\left(r\right)\;-\;\psi_{i\int }^{/}\Delta_{\int }^{-1}K_{i\int }}{\int_{0}^{1}W{\;}_{i}^{2}\;\left(r\right)\;d\;r\;-\;K_{i\int }^{/}\Delta_{\int }^{-1}K_{i\int }}$$

The present study used Pesaran and Yamagata's [91] approach for testing slope heterogeneity and Equation (8) and Equation (9) will serve the purpose.

(8) $$\bar{\Delta }=\sqrt{N}\left(\frac{N^{-1}\bar{S}-k}{\sqrt{2k}}\right)∼X_{k}^{2}$$

(9) $${\bar{\Delta }}_{\text{adj}.}=\sqrt{N}\left(\frac{N^{-1}\bar{S}-k}{v\left(T,k\right)}\right)∼N\left(0,1\right)$$

The co-integrating relationship between economic progress and its factors will be tested by using Westerlund's [92] co-integration approach and the outcomes based on Equation (10) and Equation (11) should must be significant.

(10) $$G_{t}=\frac{1}{N}\;\sum_{i=1}^{N}\left(\frac{{\hat{\lambda }}_{i}^{k}}{s.e.\left({\hat{\lambda }}_{i}^{k}\right)}\right)$$

(11) $$G_{a}=\frac{1}{N}\;\sum_{i=1}^{N}\left(\frac{T{\hat{\lambda }}_{i}^{k}}{{\hat{\lambda }}_{i}^{k}\left(1\right)}\right)\;\text{where}\;{\hat{\lambda }}_{i}^{k}\left(1\right)=\frac{{\hat{\omega }}_{\text{ui}}}{{\hat{\omega }}_{\text{yi}}}$$

$\text{and}\;{\hat{\omega }}_{\text{ui}}\;;\;{\hat{\omega }}_{\text{yi}}$ are Newey and West's [93] long-run variance estimators which further calculated with the help of Equation (12) and Equation (13).

(12) $$P_{t}=\frac{{\hat{\lambda }}_{i}^{k}}{s.e.\left({\hat{\lambda }}_{i}^{k}\right)}$$

(13) $$P_{a}=T{\hat{\lambda }}_{i}^{k}$$

To estimate the CS-ARDL model we will apply an approach established by Chudik and Pesaran [94]. Here Equation (14) and Equation (15) will help to develop a CS-ARDL model.

(14) $$\Delta {\text{lnGDPPC}}_{\text{it}}=\sum_{j=1}^{p}a_{\text{ij}}\Delta {\text{lnGDPPC}}_{i,t-j}+\sum_{j=0}^{q}a_{\text{ij}}\Delta {\text{lnLAB}}_{i,t-j}+\sum_{j=0}^{q}a_{\text{ij}}\Delta {\text{lnCAP}}_{i,t-j}+\sum_{j=0}^{q}a_{\text{ij}}\Delta {\text{lnTOU}}_{i,t-j}+\sum_{j=0}^{q}a_{\text{ij}}\Delta {\text{lnFFEC}}_{i,t-j}+\sum_{j=0}^{q}a_{\text{ij}}\Delta {\text{lnREC}}_{i,t-j}+\sum_{j=0}^{q}b_{\text{ij}}\Delta {\text{lnEXPORT}}_{i,t-j}+\sum_{j=1}^{p}b_{\text{ij}}{\text{lnGDPPC}}_{i,t-j}+\sum_{j=0}^{q}b_{\text{ij}}{\text{lnLAB}}_{i,t-j}+\sum_{j=0}^{q}b_{\text{ij}}{\text{lnCAP}}_{i,t-j}+\sum_{j=0}^{q}b_{\text{ij}}{\text{lnTOU}}_{i,t-j}+\sum_{j=0}^{q}b_{\text{ij}}{\text{lnFFEC}}_{i,t-j}+\sum_{j=0}^{q}b_{\text{ij}}{\text{lnREC}}_{i,t-j}+\sum_{j=0}^{q}b_{\text{ij}}{\text{lnEXPORT}}_{i,t-j}+\mu_{1i}+\varepsilon_{1\text{ij}}$$

(15) $$\Delta {\text{lnGDPPC}}_{\text{it}}=\sum_{j=1}^{p}c_{\text{ij}}\Delta {\text{lnGDPPC}}_{i,t-j}+\sum_{j=0}^{q}c_{\text{ij}}\Delta {\text{lnLAB}}_{i,t-j}+\sum_{j=0}^{q}c_{\text{ij}}{\text{lnCAP}}_{i,t-j}+\sum_{j=0}^{q}c_{\text{ij}}\Delta {\text{lnTOU}}_{i,t-j}+\sum_{j=0}^{q}c_{\text{ij}}\Delta {\text{lnFFEC}}_{i,t-j}+\sum_{j=0}^{q}c_{\text{ij}}\Delta {\text{lnREC}}_{i,t-j}+\sum_{j=0}^{q}c_{\text{ij}}\Delta {\text{lnEXPORT}}_{i,t-j}+\sum_{j=1}^{p}d_{\text{ij}}{\text{lnGDPPC}}_{i,t-j}+\sum_{j=0}^{q}d_{\text{ij}}{\text{lnLAB}}_{i,t-j}+\sum_{j=0}^{q}d_{\text{ij}}{\text{lnCAP}}_{i,t-j}+\sum_{j=0}^{q}d_{\text{ij}}{\text{lnTOU}}_{i,t-j}+\sum_{j=0}^{q}d_{\text{ij}}{\text{lnFFEC}}_{i,t-j}+\sum_{j=0}^{q}d_{\text{ij}}{\text{lnREC}}_{i,t-j}+\sum_{j=0}^{q}d_{\text{ij}}{\text{lnFDI}}_{i,t-j}+\mu_{2i}+\varepsilon_{2\text{ij}}$$

To check robustness, the Common Correlated Effects Mean Group (CCEMG) technique developed by Pesaran [95] will be adopted and Equation (16) and Equation (17) will be used to examine estimates of AMG and CCEMG

(16) $$y_{\text{it}}=\alpha_{i}+b_{i}^{/}x_{it}+c_{i}^{t}+d_{i}{\hat{\mu }}_{t}^{*}+e_{it}=>{\hat{b}}_{AMG}=N^{-1}\sum_{i}{\hat{b}}_{i}$$

(17) $$y_{\text{it}}=\alpha_{\text{it}}+\beta_{i}x_{it}+\lambda_{i}h\left(\bar{\lambda }f_{i}\right)+u_{\text{it}}$$

The one-year stochastic term with negative sign and statistical significance are necessary conditions for achieving stable and long-run equilibrium [[96], [97], [98], [99], [100]]. Here, Equation (18) and Equation (19) will help to obtain short-run coefficients

(18) $$\Delta {\text{lnGDPPC}}_{\text{it}}=\sum_{j=1}^{p}f_{\text{ij}}\Delta {\text{lnGDPPC}}_{i,t-j}+\sum_{j=0}^{q}f_{\text{ij}}\Delta {\text{lnLAB}}_{i,t-j}+\sum_{j=0}^{q}f_{\text{ij}}\Delta {\text{lnCAP}}_{i,t-j}+\sum_{j=0}^{q}f_{\text{ij}}\Delta {\text{lnTOU}}_{i,t-j}+\sum_{j=0}^{q}f_{\text{ij}}\Delta {\text{lnFFEC}}_{i,t-j}+\sum_{j=0}^{q}f_{\text{ij}}\Delta {\text{lnREC}}_{i,t-j}+\sum_{j=0}^{q}f_{\text{ij}}\Delta {\text{lnEXPORT}}_{i,t-j}+\gamma_{1,\text{ij}}\;{\text{ECM}}_{i,t-1}+\eta {\;}_{1,\text{ij}}$$

(19) $$\Delta {\text{lnGDPPC}}_{\text{it}}=\sum_{j=1}^{p}\;g_{\text{ij}}\Delta {\text{lnGDPPC}}_{i,t-j}+\sum_{j=0}^{q}g_{\text{ij}}\Delta {\text{lnLAB}}_{i,t-j}+\sum_{j=0}^{q}g_{\text{ij}}{\text{lnCAP}}_{i,t-j}+\sum_{j=0}^{q}g_{\text{ij}}\Delta {\text{lnTOU}}_{i,t-j}+\sum_{j=0}^{q}g_{\text{ij}}\Delta {\text{lnFFEC}}_{i,t-j}+\sum_{j=0}^{q}g_{\text{ij}}\Delta {\text{lnREC}}_{i,t-j}+\sum_{j=0}^{q}g_{\text{ij}}\Delta {\text{lnEXPORT}}_{i,t-j}+\gamma_{2,\text{ij}}\;{\text{ECM}}_{i,t-1}+\eta {\;}_{2,\text{ij}}$$

To test the causal relationship between dependent and independent variables in heterogeneous panels, we will apply the procedure proposed by Dumitrescu and Hurlin [101]. The null hypothesis of no homogeneous causal relation running from one variable to another will be tested by using W-statistics and Z-bar statistics and presented in Equation (20) and Equation (21).

(20) $$W{\;}_{N,T}^{\text{HNC}}=\left(\frac{1}{N}\right)\;\sum_{i=1}^{N}W_{i,T}\;\text{Where}\;T,N\;\to \infty$$

(21) $$\tilde{Z}{\;}_{N,T}^{\text{HNC}}=\sqrt{\frac{N}{2\;x\;K}\;x\;\frac{\left(T\;-\;4\right)}{\left(T+K\;-\;2\right)}\;}x\;\left[\left(\frac{\left(T\;-\;2\right)}{T}\right)\;W{\;}_{N,T}^{\text{HNC}}\;-\;K\right]$$

The above-mentioned econometric framework is given in Fig. 1, and the results are calculated in the subsequent section.

RETRACTED

**Fig. 1:** Econometric framework.

## 4 Results and discussion

We will initiate by presenting a discussion on a statistical summary of the variables given in Table 2.

**Table 2:** Statistical summary.

**Variables**	**Mean**	**Std.** **Deviation**	**Maximum**	**Minimum**	**Skewness**	**Kurtosis**	**Sample Size**
${\text{lnGDPPC}}_{\;\text{it}}$	10.522	0.465	11.652	8.917	−0.635	3.953	930
${\text{lnLAB}}_{\text{it}}$	1.568	0.141	1.893	1.197	0.012	2.922	930
${\text{lnCAP}}_{\text{it}}$	3.139	0.193	4.002	2.387	−0.030	4.723	930
${\text{lnTOU}}_{\text{it}}$	1.622	0.136	1.920	1.317	0.237	2.299	930
${\text{lnFFEC}}_{\;\text{it}}$	6.171	1.493	10.068	3.381	0.362	2.721	930
${\text{lnREC}}_{\;\text{it}}$	0.259	0.150	0.460	−0.503	−1.089	4.971	930
${\text{lnEXPORT}}_{\;\text{it}}$	0.368	0.064	0.543	0.218	0.348	3.416	930
${\text{lnFDI}}_{\;\text{it}}$	0.009	0.015	0.0047	−0.072	−1.149	7.166	930

The values of standard deviation for GDP, labor force, capital formation, tourism, fossil fuel energy, renewable energy, and exports are found less than their corresponding mean values therefore, we may conclude that all these stated variables are under-dispersed. This confirms that the required number of outliers for a normal distribution meets the criterion therefore, we may conclude that all variables have normal distributions, however, FDI is over-dispersed therefore it is not normally distributed.

After discussing the statistical summary, now variance inflation factor (VIF) will be calculated for inspecting the presence of multicollinearity between the independent variables of the study. Table 3 depicts the value of VIF, according to Asteriou and Hall [102], if the VIF value is witnessed as less than 10 then there is no multicollinearity. The result of VIF reveals a weak correlation of dependent variables with the other explanatory variables considered in this study hence we may conclude that all the explanatory variables are strictly exogenous within the selected functional forms. The results are provided below in Table 3.

**Table 3:** Correlation Matrix (VIF values).

**Variables**	${\text{lnLAB}}_{\text{it}}$	${\text{lnCAP}}_{\text{it}}$	${\text{lnTOU}}_{\text{it}}$	${\text{lnFFEC}}_{\;\text{it}}$	${\text{lnREC}}_{\;\text{it}}$	${\text{lnEXPORT}}_{\;\text{it}}$	${\text{lnFDI}}_{\;\text{it}}$
${\text{lnLAB}}_{\text{it}}$	–						
${\text{lnCAP}}_{\text{it}}$	1.003	–					
${\text{lnTOU}}_{\text{it}}$	1.850	1.039	–				
${\text{lnFFEC}}_{\;\text{it}}$	9.510	1.001	1.658	–			
${\text{lnREC}}_{\;\text{it}}$	1.003	1.032	1.005	1.035	–		
${\text{lnEXPORT}}_{\;\text{it}}$	1.903	1.003	1.129	1.486	1.024	–	
${\text{lnFDI}}_{\;\text{it}}$	1.213	1.000	1.022	1.124	1.013	1.648	–

Besides this, CD is also found in data series by using the method proposed by Pesaran [89]. From Table 4 we may see that the null hypothesis of CD is rejected as the probability value of the CD-test for all the variables is witnessed as significant. Therefore, we conclude the presence of CD in our study.

RETRACTED

**Table 4:** Results of CD test.

**Variables**	**CD Test**	**P-Values**
${\text{lnGDPPC}}_{\;\text{it}}$	105.814	0.000
${\text{lnLAB}}_{\text{it}}$	57.949	0.000
${\text{lnCAP}}_{\text{it}}$	15.101	0.000
${\text{lnTOU}}_{\text{it}}$	60.483	0.000
${\text{lnFFEC}}_{\;\text{it}}$	24.837	0.000
${\text{lnREC}}_{\;\text{it}}$	36.669	0.000
${\text{lnEXPORT}}_{\;\text{it}}$	65.272	0.000
${\text{lnFDI}}_{\;\text{it}}$	26.974	0.000

After confirmation of CD, the application of the first generation unit root test turns redundant therefore, we are using CIPS and CADF tests which are suitable if data series suffer from CD issues. For the variables that have unit roots, the CIPS-test and CADF-test values will be lower than the threshold value. In the case of the CADF test, a significant p-value of the t-bar test indicates the rejection of the null hypothesis as given in Table 5.

**Table 5:** Panel unit root test.

**Variables**	**CIPS-Stats**	**CADF-Test**	**Variables**	**CIPS-Stats**	**CADF-Test**
${\text{lnGDPPC}}_{\;\text{it}}$	−1.996	−1.805 (0.419)	$\Delta {\text{lnGDPPC}}_{\;\text{it}}$	−3.941	−3.063 (0.000)
${\text{lnLAB}}_{\text{it}}$	−1.954	−1.845 (0.330)	${\Delta \text{lnLAB}}_{\text{it}}$	−3.813	−3.797 (0.000)
${\text{lnCAP}}_{\text{it}}$	−2.142	−2.105 (0.025)	${\Delta \text{lnCAP}}_{\text{it}}$	−4.704	−3.791 (0.000)
${\text{lnTOU}}_{\text{it}}$	−2.047	−1.897 (0.229)	${\Delta \text{lnTOU}}_{\text{it}}$	−4.282	−2.191 (0.007)
${\text{lnFFEC}}_{\;\text{it}}$	−2.007	−1.969 (0.123)	$\Delta {\text{lnFFEC}}_{\;\text{it}}$	−4.879	−3.949 (0.000)
${\text{lnREC}}_{\;\text{it}}$	−2.398	−2.453 (0.000)	$\Delta {\text{lnREC}}_{\;\text{it}}$	−5.292	−5.476 (0.000)
${\text{lnEXPORT}}_{\;\text{it}}$	−2.013	−1.862 (0.295)	$\Delta {\text{lnEXPORT}}_{\;\text{it}}$	−3.961	−3.429 (0.000)
${\text{lnFDI}}_{\;\text{it}}$	−3.83	−2.761 (0.000)	$\Delta {\text{lnFDI}}_{\;\text{it}}$	−6.044	−5.044 (0.000)

From Table 5, we may see that the values of the CIPS-test for natural log of capital, renewable energy, and FDI remain less than critical values at level, while CADF-test values for the same variables are found to be significant, therefore; these three variables are level-stationary while other are difference-stationary. Thus CIPS test represents, that the proposed model has variables with mixed order of integration.

RETRACTED

After testing unit root now we are presenting Westerlund's [92] cointegration test and it also provides efficient estimates if the data series have CD issues. The significant “Pa” test in model-1 and significant “Ga” test in model-2 provide us evidence of the cointegrating in the data series of selected economies. as given in Table 6.

**Table 6:** Test for Co-integration.

**Test Statistics**	**Model – 1**	**Model – 2**
	**Z-Stats [P-Value]**	**Z-Stats [P-Value]**
$G_{t}$	4.932 (1.000)	4.423 (1.000)
$G_{a}$	1.243 (0.893)	−1.350 (0.089)
$P_{t}$	7.259 (1.000)	8.822 (1.000)
$P_{a}$	−3.012 (0.001)	−0.893 (0.186)

If the data series suffers from CD, it does not allow the slope of regression coefficients to remain homogeneous therefore before we estimate the results, there is a need to confirm whether the slopes of the regression coefficients are homogeneous or not by utilizing the Pesaran and Yamagata [91] test. From Table 7, we may see that significant values of ‘Δ’ and adjusted ‘Δ’ that endorse the slopes in our conceptualized functional forms are heterogeneous. The empirical results are shared below.

**Table 7:** Slope heterogeneity test.

**Modelscc/Tests**	**Δ (P-Value)**	**Adjusted Δ (P-Value)**
1st Model	21.675 (0.00)	25.163 (0.00)
2nd Model	23.154 (0.00)	26.880 (0.00)

The persistence of CD and in the case of heterogeneous slop parameters, Chudik and Pesaran [94] suggest the CS-ARDL regression. The results of CS-ARDL to determine long-run coefficients are presented in Table 8.

**Table 8:** Long run results.

**Dependent Variable**$\Delta {\text{lnGDPPC}}_{\text{it}}$		
**Variables**	**Coefficients [P-Value]**	**Coefficients [P-Value]**
${\text{lnLAB}}_{\text{it}}$	−0.774 [0.490]	−1.669 [0.259]
${\text{lnCAP}}_{\text{it}}$	0.182 [0.000]	0.190 [0.0000]
${\text{lnTOU}}_{\text{it}}$	0.641 [0.043]	0.618 [0.021]
${\text{lnFFEC}}_{\;\text{it}}$	0.135 [0.000]	0.139 [0.002]
${\text{lnREC}}_{\;\text{it}}$	0.145 [0.072]	0.190 [0.088]
${\text{lnEXPORT}}_{\;\text{it}}$	0.506 [0.076]	–
${\text{lnFDI}}_{\;\text{it}}$	–	0.334 [0.064]
F Test [P-Value]	4.16 [0.00]	3.59 [0.00]
CD Test [P-Value]	−0.74 [0.456]	−0.79 [0.428]

From Table 8, we may see that the use of unclean energy is significantly enhancing economic progress in both specifications, in the long-run period. The results depict that a one percent increase in the usage of fossil fuel energy will significantly increase economic progress by 0.13 percent according to model 1, while it will increase economic progress by 0.14 percent following model 2. The effect of fossil fuel to improve economic progress is slightly stronger in Model 2 as compared to Model 1. This finding is consistent with Gozgor et al. [63], Singh et al. [65], Le et al. [66], Syzdykova et al. [77], Asiedu et al. [10], and Asif et al. [78]. The results depict that fossil fuel is a significant factor that is playing a positive role in enhancing the economic progress of developed economies. Indirectly, such findings show that the developed economies need to understand the negative impact on the environment and need to ensure such policies which may prove helpful to attain green growth by substituting fossil fuels energy with clean energy to uplift the curve of production function. After this, we may see the coefficient of renewable energy which also appeared positive and statistically significant. This means if environmentally friendly energy is promoted in the selected developed economies then it can accelerate economic progress among the selected 30 developed economies and help them to achieve the sustainable and green growth targets. If the utilization of renewable energy increases by one percent, then it will boost economic progress by 0.14 percent in model-1 and 0.19 percent in model-2 respectively. The effect of renewable energy in Model 2 is a little stronger as compared to Model 1. Our results for renewable energy are inconsistent with the findings of Amri [61], Appiah et al. [45], and Ozturk et al. [11] who reported a negative influence of renewable energy on economic progress. As the selected 30 economies in the study are developed countries, therefore, these are capital-rich economies. The influence of the labor force appears insignificant while the influence of capital accumulation is positive and significant. This means that in capital-rich countries when they specialize in the production of capital-intensive products then economic progress in such economies expands significantly. One percent increase in the capital stock will significantly increase economic progress by 0.1824 percent in model 1 and 0.1901 percent in model 2. The effect of capital stock on economic progress is also witnessed as slightly strong in model 2 as compared to model 1. The significant coefficient of capital stock is supported by Bhattacharya et al. [58], Kahia et al. [13], Ntanos et al. [62], Pegkas [67], Fu et al. [76], and Wang et al. [79]. The capital-rich economies do not pay much attention to the usage of labor-intensive techniques of production due to increasing opportunity costs therefore; the labor force is an insignificant driver of economic progress in developed economies. The results of Pao et al. [57] and Ozturk et al. [11] also reported a negative effect of the labor force on economic progress.

RETRACTED

After this, the results further expose that tourism development is another important driver that fosters economic progress in developed economies in the long run. One percent improvement in the tourism sector is significantly expanding economic progress by 0.6407 percent as depicted in model 1 and by 0.6182 percent according to the results of model 2. More expansion in the tourism industry will enhance the inflow of resources and improve funds for more investments and expansion activities in the selected developed countries. Hence it will help in boosting production activities. The outcomes are consistent with the research of Bulgan et al. [23], Rehman et al. [28], Menyari [25], Rasool et al. [29], Luo et al. [103]and Sokhanvar and Jenkins [30]. Moreover, the study also captures the effects of exports on economic progress for testing the hypothesis of export-led growth for the selected developed economies. From the results, we may see that exports are significantly enhancing economic progress and a one percent addition in exports is significantly stimulating economic progress by 0.5066 percent. Thus the results confirm the notion of the export-led growth hypothesis for the selected developed economies. These results are in alignment with Haseeb et al. [38], Ahmad et al. (2017), Canbay [40], Li et al. [104] and Logun [83] but it is not in alignment with the results of Sultanuzzaman et al. [82]. The results further demonstrate that the inflow of FDI is significantly elevating economic progress. One percent expansion in an inflow of FDI significantly boosts economic activities by 0.3348 percent. This reveals the positive spillover effects of FDI on economic progress and confirms the results of Appiah et al. [45], Kalai and Zghidi [46], Fan et al.[105] and Worku [48] but opposing the results of Olayungbo and Quadri [43] and Ciobanu [42]. Therefore, our results are contradicting the findings of these studies. The results are robust to CD issues and the overall CS-ARDL model for the long run is the best fit. After this, to inquire about robustness, we have further employed AMG and CCEMG estimators as presented in Table 9.

**Table 9:** Robustness check for the long run coefficients.

Dependent Variable $\Delta {\text{lnGDPPC}}_{\text{it}}$				
**Variables**	**AMG**	**CCEMG**	**AMG**	**CCEMG**
${\text{lnLAB}}_{\text{it}}$	0.335 [0.752]	−0.311 [0.792]	0.416 [0.663]	−0.406 [0.748]
${\text{lnCAP}}_{\text{it}}$	0.151 [0.000]	0.168 [0.000]	0.152 [0.000]	0.181 [0.000]
${\text{lnTOU}}_{\text{it}}$	0.099 [0.102]	0.362 [0.000]	0.116 [0.040]	0.285 [0.022]
${\text{lnFFEC}}_{\;\text{it}}$	0.183 [0.000]	0.108 [0.000]	0.159 [0.000]	0.138 [0.000]
${\text{lnREC}}_{\;\text{it}}$	0.277 [0.000]	0.071 [0.146]	0.343 [0.000]	0.183 [0.053]
${\text{lnEXPORT}}_{\;\text{it}}$	0.201 [0.386]	0.160 [0.522]	–	–
${\text{lnFDI}}_{\;\text{it}}$	–	–	0.344 [0.043]	0.237 [0.032]
CDP	0.771 [0.000]	–	0.748 [0.000]	
Constant	7.512 [0.000]	−0.427 [0.893]	7.438 [0.000]	−0.903 [0.782]
Wald Test [P-Value]	104.53 [0.00]	94.24 [0.00]	90.29 [0.00]	89.19 [0.00]
CD Test [P-Value]	1.048 [0.294]	0.840 [0.401]	1.008 [0.313]	0.159 [0.873]

Note: P-values are presented in parentheses.

RETRACTED

The results presented in above Table 9 advocate the long-run coefficients of the CS-ARDL model. The coefficient of exports appeared insignificant with the correct sign. The coefficient of tourism and the coefficient of renewable energy are witnessed as insignificant in one out of four cases. The coefficients of the common dynamic process in the output of the AMG estimator are witnessed as positive and statistically significant. This means that the role of unobserved or heterogeneous factors at the regional or international level may significantly accelerate economic progress in the selected 30 developed economies. The diagnostics of Table 9 are also in alignment with the diagnostics of Table 8. From the results of Table 10, we may see that the use of nonrenewable energy is significantly playing a crucial role in stimulating economic progress in the short run in developed economies. This finding is similar to the finding in the long run. If we look at the coefficients, we may say that economic progress increases by 0.1172 percent according to model 1 and by 0.1313 percent according to model 2, as a result of a one percent expansion in the use of nonrenewable in the short run in the selected sample economies. In the long run, the response of economic progress toward the use of renewable energy remains statistically significant. One percent increase in renewable energy will increase economic progress by 0.1349 percent in model 1 and 0.1568 percent in model 2. These results are also in alignment with the long-run results. The results are presented in Table 10.

**Table 10:** Short run coefficients.

Dependent Variable $\Delta {\text{lnGDPPC}}_{\text{it}}$		
**Variables**	**Variables**	**Variables**
$\Delta {\text{lnGDPPC}}_{\;\text{it}\;-\;2}$	0.106 [0.006]	0.105[0.005]
${\text{lnLAB}}_{\text{it}}$	−0.603 [0.565]	−1.202 [0.330]
${\text{lnCAP}}_{\text{it}}$	0.160 [0.000]	0.160 [0.000]
${\text{lnTOU}}_{\text{it}}$	0.465 [0.050]	0.448 [0.021]
$\Delta {\text{lnFFEC}}_{\;\text{it}}$	0.117 [0.000]	0.131 [0.000]
$\Delta {\text{lnREC}}_{\;\text{it}}$	0.135 [0.044]	0.157 [0.088]
$\Delta {\text{lnEXPORT}}_{\;\text{it}}$	0.371 [0.078]	–
$\Delta {\text{lnFDI}}_{\;\text{it}}$	–	0.277 [0.084]
${\text{ECM}}_{\;t\;-\;1}$	−0.894 [0.000]	−0.895 [0.000]

The findings further expose that the labor force reports an insignificant impact on economic progress while capital stock significantly accelerates economic progress respectively. One percent increase in capital stock is significantly accelerating economic progress by 0.1605 percent in model 1 and 0.1602 percent in model 2. This finding is also in alignment with the findings in the long run. Besides this, tourism development, exports, and inflow of FDI are significantly expanding economic progress in the selected developed economies in the short run. One percent increase in tourism development is increasing economic progress by 0.4650 percent in model 1 and 0.4483 percent in model 2 in the short run. Similarly, by expanding exports by one percent, economic progress is significantly stimulated by 0.3711 percent and due to a one percent increase in the inflow of FDI significantly elevates economic progress by 0.2775 percent in the short run respectively.

RETRACTED

The coefficient of the second period lagged per capita GDP is significantly boosting the economic progress of the present time in the short run in both specifications. This shows that the efforts made by the government in the past years in the selected economies will help stimulate production activities in the current year. Besides this, the one-year lagged stochastic term is also witnessed as negative and significant which confirms the convergence to achieve equilibrium. The speed of adjustment for achieving long-run equilibrium in model 1 is witnessed as 89.39 percent in model 1 while it is 89.51 percent in model 2. The selected economies will achieve long-run equilibrium in about 1.12 years in both specifications.

After explaining short-run coefficients, this study further tests the directional causal relation between the selected variables in the heterogeneous panel case by applying the method proposed by Dumitrescu and Hurlin [101]. The causal relation for model 1 is presented in Table 11 while the causal relation for model 2 is reported in Table 12 respectively.

**Table 11:** Panel causality tests for model 1.

$W{\;}_{N,T}^{\text{HNC}}\;-\;\text{Stats}$							P−Values							
$\tilde{Z}{\;}_{N,T}^{\text{HNC}}\;-\;\text{Stats}$														
**Variables**	$\Delta {\text{lnGDPPC}}_{\;\text{it}}$		$\Delta {\text{lnLAB}}_{\;\text{it}}$		$\Delta {\text{lnCAP}}_{\;\text{it}}$		$\Delta {\text{lnTOU}}_{\;\text{it}}$		$\Delta {\text{lnFFEC}}_{\;\text{it}}$		$\Delta {\text{lnREC}}_{\;\text{it}}$		$\Delta {\text{lnEXPORT}}_{\;\text{it}}$	
$\Delta {\text{lnGDPPC}}_{\;\text{it}}$	–		2.40	0.00	3.70	0.00	1.47	0.19	2.20	0.00	1.14	0.84	2.34	0.00
			4.44		8.82		1.31		3.76		0.20		4.25	
$\Delta {\text{lnLAB}}_{\;\text{it}}$	8.11	0.00	–		3.00	0.00	2.82	0.00	4.48	0.00	2.32	0.00	5.25	0.00
	23.71				6.48		5.85		11.46		4.19		14.06	
$\Delta {\text{lnCAP}}_{\;\text{it}}$	3.42	0.00	2.54	0.00	–		2.33	0.00	1.78	0.02	1.73	0.03	2.49	0.00
	7.89		4.91				3.88		2.37		2.18		4.75	
$\Delta {\text{lnTOU}}_{\;\text{it}}$	1.22	0.65	1.59	0.08	1.34	0.39	–		1.72	0.03	2.28	0.00	1.28	0.51
	0.46		1.74		0.86				2.14		4.03		0.66	
$\Delta {\text{lnFFEC}}_{\;\text{it}}$	2.71	0.00	3.68	0.00	1.79	0.02	2.59	0.02	–		1.50	0.15	2.28	0.00
	5.50		8.76		2.38		5.10				1.43		4.03	
$\Delta {\text{lnREC}}_{\;\text{it}}$	2.42	0.00	3.12	0.00	2.52	0.00	2.45	0.00	2.49	0.00	–		1.67	0.05
	4.51		6.89		4.85		4.63		4.76				1.99	
$\Delta {\text{lnEXPORT}}_{\;\text{it}}$	2.56	0.00	2.05	0.00	4.64	0.00	2.14	0.00	1.37	0.33	2.63	0.00	–	
	4.99		3.26		12.01		3.59		0.97		5.21

RETRACTED

**Table 12:** Panel causality tests for model 2.

$W{\;}_{N,T}^{\text{HNC}}\;-\;\text{Stats}$							P−Values							
$\tilde{Z}{\;}_{N,T}^{\text{HNC}}\;-\;\text{Stats}$														
**Variables**	$\Delta {\text{lnGDPPC}}_{\;\text{it}}$		$\Delta {\text{lnLAB}}_{\;\text{it}}$		$\Delta {\text{lnCAP}}_{\;\text{it}}$		$\Delta {\text{lnTOU}}_{\;\text{it}}$		$\Delta {\text{lnFFEC}}_{\;\text{it}}$		$\Delta {\text{lnREC}}_{\;\text{it}}$		$\Delta {\text{lnFDI}}_{\;\text{it}}$	
$\Delta {\text{lnGDPPC}}_{\;\text{it}}$	–		2.40	0.00	3.70	0.00	1.47	0.19	2.20	0.00	1.14	0.84	2.04	0.00
			4.44		8.82		1.31		3.76		0.20		3.25	
$\Delta {\text{lnLAB}}_{\;\text{it}}$	8.11	0.00	–		3.00	0.00	2.82	0.00	4.48	0.00	2.32	0.00	1.84	0.01
	23.71				6.48		5.85		11.46		4.19		2.56	
$\Delta {\text{lnCAP}}_{\;\text{it}}$	3.42	0.00	2.54	0.00	–		2.33	0.00	1.78	0.02	1.73	0.03	1.48	0.18
	7.89		4.91				3.88		2.37		2.18		1.34	
$\Delta {\text{lnTOU}}_{\;\text{it}}$	1.22	0.65	1.59	0.08	1.34	0.39	–		1.72	0.03	2.28	0.00	1.34	0.38
	0.46		1.74		0.86				2.14		4.03		0.88	
$\Delta {\text{lnFFEC}}_{\;\text{it}}$	2.71	0.00	3.68	0.00	1.79	0.02	2.59	0.02	–		2.81	0.00	0.83	0.39
	5.50		8.76		2.38		5.10				5.85		−0.86	
$\Delta {\text{lnREC}}_{\;\text{it}}$	2.42	0.00	3.12	0.00	2.52	0.00	2.45	0.00	2.49	0.00	–		1.11	0.92
	4.51		6.89		4.85		4.63		4.76				0.10	
$\Delta {\text{lnFDI}}_{\;\text{it}}$	3.41	0.00	2.64	0.00	1.63	0.07	2.02	0.00	1.37	0.33	0.98	0.72	–	
	7.84		5.28		1.84		3.16		0.97		−0.35			

From above Table 11, we may see that the estimated results of W-stats and Z-bar stats for model 1 confirm the bidirectional association of the labor force with economic progress, between capital formation and economic progress, between nonrenewable energy and economic progress, and between exports and economic progress. The presence of unidirectional causal relation is witnessed from economic progress to renewable energy for model 1. The empirical results presented in Table 11 for Model 2 also confirm the bidirectional relation between economic progress and labor force, between economic progress and capital formation, between nonrenewable energy and economic progress, and between the inflow of FDI and economic progress. However, unlike model 1, for model 2, the study discloses the presence of unidirectional relation which is running from economic progress to renewable energy in the selected developed economies. This discussion allows us to confirm the feedback effect hypothesis, and also endorse the economic progress and the energy conservation hypothesis for model 1 and model 2. The finding of the feedback hypothesis is consistent with Satti et al. [7] while the finding of the conservation hypothesis is supported by Bekun and Agboola [6]. The results for model 2 are reported in the following Table 12.

RETRACTED

## 5 Conclusion and policy implication

The purpose of this research is to inspect the influence of nonrenewable energy and renewable energy on the economic progress of the 30 selected developed economies. After utilizing the CS-ARDL approach over the annual sample period from 1990 to 2020, this study concludes that the utilization of both renewable energy and nonrenewable energy significantly accelerates economic progress in the selected 30 developed economies. The results further confirm that the expansion of tourism development, enhancing capital-intensive methods of production, increasing exportable items, and boosting the inflow of FDI are significantly strengthening production activities and hence economic progress in developed economies. Moreover, this study also confirms the presence of a feedback effect between nonrenewable energy and economic progress in both models while economic progress is found in causing renewable energy in both models hence energy conservation hypothesis stands valid for this case. The causal relation also confirms the presence of a bidirectional relation between the labor force and economic progress, between capital stock and economic progress, between exports and economic progress, and between the inflow of FDI and economic progress in the selected sample economies.

Based on these findings, the present study proposes that renewable energy should be targeted in such a way that it can help leave its significant attributes upon economic progress. There is a need to introduce incentives for those industries producing goods by adopting clean energy and through environmentally friendly methods, this will develop a healthy industrial competition and expedite the transition process from fossil fuels to clean energy-based production procedures at macro and micro levels. Although fossil fuel energy helps expand economic progress we believe it will also harm the environmental quality. The empirical results suggest that targeting nonrenewable energy should be made carefully as if it is reduced, it will reduce economic progress and in turn, the slow pace of economic progress will adversely influence the promotion of renewable energy. Moreover, a careful attempt through which emphasis may be shifted from nonrenewable energy to renewable energy in such a way that it should not harm economic progress. Otherwise, it will not allow clean energy to deliver fruitful results for improving economic progress in the light of improved environmental quality. Moreover, the positive role of tourism development, exports, FDI, and capital formation also allows us to suggest that these are the potential drivers that are helping in enhancing production activities, and therefore, these should be diversified enough that they can further give stimulus to the production function of the selected economies. These policy implications aim to create an enabling environment that harnesses the positive impacts of clean energy, tourism development, exports, and FDI inflow on economic growth, fostering a more sustainable and equitable future. However, the findings of this study are limited by the data range, use of controlling factors, and methodology used in this particular study. Additionally, incorporating further control variables and considering other important monetary factors such as interest rates, the quality of institutions, taxes on the energy sector, and consideration of export facilitation schemes could provide deeper insights into the issue of stagnant economic growth.

RETRACTED

## Data availability statement

The data used in the manuscript will be available on request.

## CRediT authorship contribution statement

**Hunag Chenhui:** Writing – review & editing, Writing – original draft, Formal analysis, Data curation. **Muhammad Shahid Hassan:** Writing – original draft, Data curation, Conceptualization. **Sahar Afshan:** Writing – review & editing, Software, Methodology. **Imran Hanif:** Writing – review & editing, Methodology, Investigation. **Muhammad Umair:** Software, Investigation, Data curation, Conceptualization. **Olayan Albalawi:** Writing – review & editing, Methodology, Formal analysis.

## Declaration of competing interest

The authors declare the following financial interests/personal relationships which may be considered as potential competing interests:Imran Hanif reports statistical analysis and writing assistance were provided by Government College University Lahore Pakistan.Imran Hanif reports a relationship with Heliyon Elsevier that includes: board membership. We have no conflict of interest to disclose here. If there are other authors, they declare that they have no known competing financial interests or personal relationships that could have appeared to influence the work reported in this paper.

RETRACTED

## Figures and Tables

**(a):** List of the Selected Developed Economies

Australia	Greece	New Zealand
Austria	Hungary	Norway
Belgium	Ireland	Poland
Canada	Italy	Portugal
Chile	Japan	Singapore
Denmark	Korea, Rep.	Spain
Estonia	Latvia	Sweden
Finland	Lithuania	Switzerland
France	Luxembourg	United Kingdom
Germany	Netherlands	United States
